# Portable Face-Shielding Device Based on sEMG Considering the COVID-19 Scenario

**DOI:** 10.1155/2023/8231073

**Published:** 2023-07-08

**Authors:** Tian Lyu, Dong Yang Liu, Chen Shao, ZiJie Zhang

**Affiliations:** ^1^School of Mechatronics Engineering, Beijing Institute of Technology, 100081 Beijing, China; ^2^Physics and Astronomy (PHYSX), Cardiff University, CF24 3AA, UK; ^3^School of Mechanical Engineering, Xi'an Jiaotong University, Xi'an 710049, China; ^4^City University of Hong Kong, Hong Kong 999077, Hong Kong

## Abstract

Wearing a mask greatly reduced the possibility of infection during the COVID-19 pandemic. However, major inconveniences occur regarding patients with upper limb amputations, as they cannot independently wear masks. As a result, bacterial contamination is caused by medical staff touching the quilt when helping. Furthermore, this effect can occur with ordinary people due to accidental touch. This research aims to design an automatic and portable face shield assistive device based on surface electromyography (sEMG) signals. A concise face shield-wearing mechanism was built through 3D printing. A novel decision-making control method regarding a feature extraction model of 16 signal features and a Softmax classification neural network model were developed and tested on an STM32 microcontroller unit (MCU). The optimized electrode was fabricated using a carbon nanotube (CNT)/polydimethylsiloxane (PDMS). The design was further integrated and tested, showing a promising future for further implementation.

## 1. Introduction

In recent years, the COVID-19 epidemic has been rampant. As a result, face shielding has been effectively used to avoid the spread of the corresponding virus [1]. In the absence of a shelter-in-place strategy, infections, hospitalizations, and deaths were reduced by 37.7%, where the interquartile range (IQR) was 36.1–39.4%, 44.2% (IQR: 42.9–45.8%), and 47.2% (IQR: 45.5–48.7%), respectively, as nonmedical masks were worn by 75% of the population reduced [2]. The use of general facemasks has significant benefits, especially if they are adopted earlier, and at least some benefit is realized across a range of epidemic intensities. Furthermore, masks can be used in addition to other interventions, such as social distancing and hygienic measures, ultimately resulting in a nonlinear decrease in epidemic mortality and healthcare system burden [3]. During the COVID-19 outbreak, many new developments related to healthcare utilized electromyography (EMG) or electroencephalogram (EEG). Setiawan et al. proposed a stroke rehabilitation monitoring method using EEG [4], Bano and Hussain could identify patients that were infected by COVID-19 using the EMG technique [5], and L. Jiang et al. developed an advising device for at-home exercise using sEMG [6].

Some disabled and paralyzed patients, however, who have both arms amputated cannot wear face masks independently. According to the latest survey reported by China Disabled Persons' Federation, in 2010, China had 20.54 billion amputation patients [7], of which 2/3 were upper limb amputees [8]. In addition, there is a nonnegligible group that has a severe impairment of both upper-and triple-limb functions [9]. However, assistance in public places increases the risk of viral infection. Furthermore, cross-infection in hospitals when nurses take care of paralyzed patients and manually wear face shields can also occur. [10] Nevertheless, patients who cannot or have difficulties putting on masks by themselves arrive at hospitals without wearing masks or need to call a nurse for assistance at their home. As a result, the person can get infected if the nurse or people in the hospital are recessive carriers of COVID-19. Many casual activities, such as dining and drinking, require that masks are constantly put on and off. However, some patients cannot be assisted by nurses all day. In some public places, directly touching the inside of a face shield by hand can contaminate this equipment, reducing its protection against infectious diseases and threatening health. We also believe that a new hand-controlled face-shielding device could be convenient for ordinary people. Hence, a noncontact wearable face-shielding-wearing system is proposed.

Heckendorn [11] and Backers Today [12] separately developed two automated face-shielding-wearing systems controlled through buttons. The automatic face shielding of Heckendorn is promising due to its mechanical structure and portability. Furthermore, the one designed by Backers Today is convenient for drinking water. These designs, therefore, reduce the possibility of contaminating face shields and are conducive for people with disabilities.

Huang developed an automask utilizing an ultrasonic sensor and an sEMG sensor that allowed the wearer to actuate when sneezing by contracting the abdominal muscle while manually covering the ultrasonic sensor [13]. This design could detect and avoid the sneeze spreading; however, the situations in which such devices can be applied are limited. Furthermore, the mask is not suitable for patients with upper limb amputations, as it can only be actuated by contracting the abdominal muscle while covering the ultrasonic sensor by hand. The utilization of an HC-SR04 ultrasonic distance sensor would significantly harm the cost efficiency of the design. The HC-SR04 module is an active measurement instrument [14] that continuously emits an echo pulse at a 40 kHz frequency [15]. Owing to the active detection limit, the power consumption of the HC-SR04 module is incessant during wearing. In contrast, the sEMG module is a passive measurement instrument whose power consumption is much lower; therefore, it is more suitable for casual wearing. Moreover, the ultrasonic distance sensor can be accidentally triggered from the outer environment, such as the clothing of the user or the impact caused by passing-by pacers. Furthermore, the signals of ultrasonic distance sensors commonly fluctuate (fluctuation phenomenon) [16], even though a threshold value is set to avoid accidental triggering. In addition, the control algorithm of the design involved no signal classification, increasing the risk of accidentally triggering the mechanism. The actuation and control of the servo motor without a signal classification are usually achieved by manually setting the threshold of the triggering voltage amplitude. [15] However, unwanted spike signals that trigger the actuators can be generated. For example, accidental pressing on the sEMG sensors or external force-induced position shift of the electrodes would create spikes and noise. Furthermore, the fluctuation phenomenon of the ultrasonic distance sensors contributes to more accidental actuation in Taliyah Huang's design. Finally, controlling the mask based on the abdominal muscle is not feasible, as the body fat at a selected abdomen position significantly varies depending on the person; therefore, the EMG signal cannot be commonly applied. Different factors, such as epidermal body fat, significantly influence the sEMG measurement, [17]. As lipids easily accumulate in the abdomen, the abdominal muscle EMG could be weak to be detected when facing thick abdominal fat tissue.

To solve these problems, we designed a portable, noncontact, and automatic face-shielding-wearing device that considers the EMG signals.

## 2. Background Knowledge

An electromyography instrument is used in EMG to record muscle bioelectric signals. These electrical signals can describe some characteristic behaviors of the human muscles. EMG signals can be used in many fields, such as clinical applications [18] and human-computer interaction [19]. More direct monitoring of the human body can be achieved through the analysis, processing, classification, and various signal analysis methods of these signals [20]. New implementations of EMG, such as muscular paralysis disease prediction using EMG, have been developed during the pandemic [21].

However, people who are inconvenienced by wearing masks often need to adapt themselves to EMG devices for a long time. Commercial electrodes are generally Ag/AgCl electrodes; however, these components should be avoided, as they cause damage to human skin [22]. As a result, we used carbon nanotubes, which are nontoxic, harmless, and pollution-free [23], as the primary material for the electrode, increasing its stronger skin affinity and allowing it to be more suitable for long-term use.

The proposed device collects and analyzes the human body EMG signal, realizing thereafter, through machine learning, the wearing and removal of the face shield according to the human body EMG signal. As a result, it does not need to be manually controlled. This study used the specific location of the muscle signal of a dual-channel sEMG detector. We also improved the electrode material in contact with the human body, resulting in a more suitable material for long-term use. Based on the corresponding signal feature processing and machine learning classification, noncontact automatic face shielding and wearing could be realized.

## 3. System Architecture and Methodology

The main objective of this study was to design a portable face-shielding device based on sEMG. The user of the proposed device could wear/undress the mask by contracting two specific muscles, fulfilling the noncontact demand for paralyzed patients with amputated upper limbs or ordinary people, therefore avoiding the accidental touch of the inner surface of the face shield. By selecting two independent muscles that do not usually form a synergic pattern, the device can be precisely actuated based on the corresponding gesture, thereby avoiding accidental triggers. To realize this purpose, at least three primary components were involved: data acquisition units, portable data processing units, and automatic face-shielding mechanisms.

A data flow chart of the designed system, composed of these primary components, is shown in Figure 1. We use a 2 MyoWare™ Muscle Sensor (AT-04-001) [24] to achieve bichannel input of the sEMG signals, as the EMG signals of two independent muscles were detected. A hardware bandpass filtering circuit and rectifying and amplifying procedures were integrated into the MyoWare module. The analog sEMG signal was further converted to a digital signal through an analog to digital converter (ADC) on a STM32F103ZET6 microcontroller unit (MCU), which is a portable data processing unit. Based on the received data, our algorithm yields a decision that fulfills the user demand. Accordingly, the triggering signal is sent to the automatic face-shielding mechanism via IIC based on the corresponding gesture.

Many studies, among which the methodologies are profound examples of our research, have been conducted on implementations utilizing sEMG. References [25–28] investigated muscle selection for sEMG electrode placement or gesture selection. References [26–30] analyzed the sEMG signal preprocessing or segmentation. References [25–29] studied a feature extraction procedure of the signal and a classification method utilizing neural networks or a support vector machine (SVM), which was integrated into [25–29]. Based on the methodologies investigated, our research methodology can be summarized as indicated in Figure 2.

To increase the dermotropic property and electrical conductivity of the electrodes, we have investigated the improvement of the electrode material. The mechanical structural design targets a lightweight and conciseness compatible wearable mechanism. As shown in Figure 2, the model training of the EMG data flow can be divided into an offline data training process and a real-time model training.

In the offline model training procedure, the data were, first, preprocessed. Afterward, serial feature extraction based on the segmented data batches was conducted. The classification process was based on artificial neural networks (ANN) in this research.

Models are obtained through offline training, regardless of the real-time control of the mechanism and considering datasets stored on a personal computer (PC). Further development of these idealized models needs to be achieved and calibrated in the real-time training procedure. Their parameters were, therefore, carefully adjusted based on the actual performance of the device to achieve the optimized conditions.

Our experimental setups of the data flow model training are shown in Figure 3, which indicates the key components for the feature extraction model and the classification neural network training. The red arrows represent the power supply directions; the blue lines stand for data flows from the peripheral devices to the MCU. In contrast, the yellow arrows represent the opposite data flow. Both data flow represented by the yellow and blue arrows should be omitted during the real-time optimization to achieve the portability of the design. The green and grey arrows indicate the data flow between the MCU and peripherals.

To illustrate the hardware selection, two MyoWare™ muscle sensors (AT-04-001) were selected for the sEMG signal detection. A 32-bit microcontroller composed of an ARM Cortex-M3 core STM32F103ZET6 [31] MCU module was selected to execute the computational tasks of this portable device, owing to its computational performance and stability. A push button, which was pressed to indicate the need for the shielding mask, was used for signal labeling. A 5 V polymer battery was needed for the power supply. The PCA9685 module is a 16-channel PWM output motor control module [32]. In this study, we realized control of a FUTABA Corp. S3003 servo motor through IIC communication and PCA9685.

## 4. Design of Mechanism

The mechanical design of the face-shielding device should promote function, reliability, and economic characteristics. To achieve a functional design, the basic motion form, as well as the main measurement of the device, should be analyzed based on practical applications. After completing the overall design of the device, which is usually idealistic and abstract, its reliability must be evaluated; therefore, specific parts, such as rockers and connectors, should be selected, and mechanical calculations and analyses are necessary to ensure the feasibility of movement. Certain elements might also be modified and optimized. Finally, the material and manufacturing process are were selected based on a limited budget.

Our face-shielding device must successfully take the face shield on and off. To simplify this situation, it can be assumed that the shield is moving around a fixed point. As this is the only movement required, the device can be designed as a planar mechanism, as shown in Figure 4(a). To further simplify the system, a rigid four-bar linkage was used as the basic structure.

As the only movement of the face shield is rotation, the mechanism has only one degree of freedom (DOF). To fulfill this requirement, a parallelogram form of the four-bar linkage was used, as shown in Figure 4(b)). Based on this adaptation, the rotary motion of the driver bar at the driven bar is duplicated, therefore creating a stable parallel relationship.

The planar DOF is governed by the following equation:

(1) $$\begin{array}{c} M=3\left(L-1\right)-2J_{1}-J_{2}, \end{array}$$

where *M* is the DOF, *L* is the number of links, and *J*_1_ and *J*_2_ are the number of lower and higher pairs, respectively. In the parallelogram linkage, where one bar is already fixed, *L* = 4, *J*_1_ = 4, and *J*_2_ = 0; therefore, *M* = 1 based on equation (1). This value of DOF indicates that the four-bar linkage of the parallelogram fulfills the requirements of this study.

The concept of the planar mechanism was, thereafter, further refined into a 3D mechanism by adding two identical four-bar linkages connected by an axis, therefore completing the structure that could be fixed on the neck of the subject and achieving a rotary motion. The dimensions of the structure were based on the human face and actual movement.  Figure 5(a) demonstrates the 3D version of the device constructed through SOLIDWORKS 2020. Two bases were placed on either side of the neck of the subject, and a servo motor was installed to drive rocker1, allowing it to complete the rotary motion. The face shield was placed between connecting rod3 and rod4.

However, according to our requirements, bar2 should be fixed to restrict the DOF to one. Moreover, the joints on which the connectors should be used have not been determined yet. As the stability of the structure must be ensured during operation, the movement of the bars moving along the axle cannot be executed. As a result, based on the reliability analysis, the joints were connected by bolts and nuts, a new base was designed to restrict the movement of bar2, and the diameters of the two axles were modified to ensure the axial constraint. The optimized mechanism is shown in Figure 5(b)).

In additive manufacturing (3D printing), simulations can be directly transformed into real objects, resulting in a swift process. The simulation in SOLIDWORKS was already implemented; therefore, due to the principle of economic design, additive manufacturing was selected as our manufacturing method. The material that has been frequently used in this process is resin, as it demonstrates suitable rigidity for the rotation of light objects, such as face shields. The accuracy of this method, however, is not satisfactory yet, which may result in higher dimensional and geometric tolerances in each part.

The proposed mechanism provides, therefore, a relatively effective procedure for taking the face shield on and off without requiring a complex structure. Furthermore, the material selected for the face-shielding device is light and the rigidity against the torque generated by the servo motor is sufficient, resulting in less stress for the subjects when using the device. However, the stability of the entire mechanism is not perfect owing to its simple structure, therefore requiring future improvements. Moreover, the mechanism might wear after a long-term operation due to the lack of protection.

## 5. Improvement of the Material of the Electrode

### 5.1. Background

The standard sEMG electrode commonly used in experiments is usually composed of gold (Au), silver (Ag), or silver-silver chloride (Ag/AgCl). Ag/AgCl is the most widely used material, as it has a lower baseline-noise interface than that of the other electrodes. Most Ag/AgCl on the market is present in the form of gel, for better maneuverability. This material can also be used in the surface coating of the electrode to reduce surface impedance and improve signal quality [33].

However, Ag/AgCl electrodes have several problems. The proposed equipment must be designed considering that people can wear it for a long time; however, the long use of an Ag/AgCl electrode can easily stimulate the skin and affect the signal quality after drying [34]. As a frequent replacement of new electrode sheets and stimulation of human skin are not considered in our design, an electrode that can be worn for a long time was developed [35].

Owing to the good dispersibility of carbon nanotubes (CNTs) and the flexibility of polydimethylsiloxane (PDMS), CNT/PDMS composites are considered good flexible conductors. The nanotubes dispersed in the electrode were in good contact with each other, forming a conductive path. Conductivity tests showed that the electrical performance depends on the concentration of carbon nanotubes. Furthermore, electrode materials are safe for biomedical applications, as they are not easily affected by sweat on the surface of the human body [36].

### 5.2. Materials and Methods

#### 5.2.1. Material Parameters

The CNT used in the electrode was manufactured by Suzhou Tanfeng Tech. Inc., China. The purity and length of the carbon nanotube were over 95 wt% and 3–12 *μ*m, respectively. The multiwall CNT was manufactured through vapor deposition. PDMS was manufactured by Shenzhen Xinwei New Material Co. Ltd. by using 909 potting glue.

#### 5.2.2. Fabrication of Electrodes

The electrode was composed of an insulating layer, conductive film, and button electrode, as indicated in Figure 6.

The CNT was dispersed into the PDMS precursor (viscosity: 4000 ± 500,909-A, Xinwei New Material Co., Ltd.) and mixed through dispersion. A crosslinking agent (viscosity: 100 ± 10,909-B, Xinwei New Material Co., Ltd), whose ratio was 10 : 1, was solidified for 12 h at room temperature. When this agent could not solidify, the button electrode was embedded in the colloid and the solidification process occurred for 24 h. A 10 : 1 ratio of PDMS was used on the periphery, forming an insulating layer to facilitate contact between the electrode and the skin.  Table 1.

As shown in Table 2, the specifications of the electrode sheet must be defined to enable the usage of the equipment for a long duration. The diameter of the conductive electrode part of the CNT/PDMS electrode sheet used in the experiment was 10 mm, which is a small part of the entire electrode. The conductive electrode (main body of the electrode), whose length and width were 36.5 mm and 30.2 mm, respectively, was composed of a PDMS solid gel. The overall thickness of the electrode sheet was 2 mm.

#### 5.2.3. Electrical Test and Specification

The impedances of the electrodes were measured using an electric meter.  Table 1 shows a test comparison diagram of commercial Ag/AgCl electrodes and CNT/PDMS electrodes considering the same specifications.

The transparent material in Figure 7 is the PDMS patch, and the black component corresponds to the CNT/PDMS electrode. The button electrode was connected on top of the CNT/PDMS to obtain an electrical signal from the device.

## 6. Electrode Positioning and Muscle Selection

The muscles were selected in this study by mainly two criteria: (1) if they are independent of each other; therefore, they ought not to collaborate to execute the same gesture, to reduce the possibility of accidentally actuating the mechanism; (2) if the selected gesture pattern is easy to achieve. Furthermore, face shielding should not affect the feasibility and regularity of the selected pattern.

The position and orientation of the muscle sensor electrodes significantly affect the strength of the signal. Owing to the differential detection mode of the sensors, two detection points and a reference position should be defined. The electrodes should be placed in the middle of the muscle body and aligned with the muscle fibers [25]. Meanwhile, the reference electrode should be placed on a separate section of the body, such as the bony portion of the elbow or a nonadjacent muscle. Due to the size of the MyoWare™ muscle sensors (AT-04-001), the sensors of the system are closely positioned (C-position). As a result, the differential voltage between the two points in the middle of the muscle body could be detected [37].

Figure 8 shows the positions of the electrode placement based on the muscle. The green box indicates the correct positioning of the electrodes (midline of the muscle belly between the innervation zone and myotendinous junction) [24].

After comprehensive consideration of the two major factors affecting the positioning of the electrodes, the gesture pattern was defined based on the zygomaticus and bicipital muscle of the arm. In particular, these muscles were selected as they can be easily contracted and their gestures can be executed by different users, such as patients with upper limb amputation and ordinary people. The gesture pattern was defined as a signal trigger when both muscles simultaneously contracted. The detailed placement of the electrodes is shown in Figure 9. To preserve the accuracy and repeatability of the experiment, the contour of the electrode was marked by using a luminous pen after each test.

After attaching the electrodes to the surface of the muscles, a bichannel ADC function was completed on the MCU utilizing a timer interrupt and setting a sampling rate of 100 Hz. The sampled data were stored in an array for further processing.

## 7. Preprocessing and Feature Extraction

The preprocessing of the sEMG signal usually involves amplification [29], filtering [26, 27, 29], rectifying [26, 27], and segmentation (or windowing) [28, 38]. An instrumental amplifier, bandpass filter, and rectifying circuits were, therefore, integrated into the MyoWare™ Muscle Sensors (AT-04-001) [24]. As a result, only data segmentation could not be conducted directly by the sensor.

A fixed-length segmentation method [38] was applied in this study. The windowing length was restricted to the performance of the STM32 MCU. The coding process of the MCU was conducted using Keil MDK v5.26 Software. Only 64, 256, and 1024 points of fast Fourier transformation (FFT), which is a method to analyze the power-related characteristics of signals from the aspect of the frequency domain, were allowed on the F1 series of the STM32 [39]. Time-frequency analysis is an important key to EMG signal feature extraction [40, 41]. Due to the selected sampling rate and the requirement for a quick response, the FFT of 64 points was used in this study. To date, a windowing of 64 data points per batch has been set for feature extraction, indicating that the response time for pattern recognition is approximately 80 ms, based on a calculation machine cycle (MC).

The acquired voltage amplitude data of the two inputs and labeling data of the push button were sent from STM32F103ZET6 to the PC using a universal asynchronous receiver/transmitter (UART) and stored in text files (.txt). The files were later processed using MATLAB, as shown in Figure 10, where the vertical and horizontal axis indicates the amplitude and the timeline, respectively. The peaks in the figure are spiky as this dataset was composed of over 15000 points of data, resulting in a contraction in the horizontal display of the graph. The data sent to MATLAB were raw data that were not binned based on 64 batch sizes, as the segmentation of the data was performed via MATLAB2019a in this simulation stage.

During the feature extraction step of this study, the model was first simulated on a PC using MATLAB2019a to test the proposed concept. Afterward, the model was coded again using the C language and executed on MCU.

In this study, 16 features, of which 11 were based on the time domain and 5 on the frequency domain, were collected to analyze the binned datasets. The features based on the time domain were the integrated EMG (IEMG), mean absolute value (MAV), modified mean absolute value 1 (MMAV1) and 2 (MMAV2), mean absolute value slope (MAVS), root mean square (RMS), variance (VAR), waveform length (WL), threshold crossing (TC), Willison amplitude (WAMP), and simple square integral (SSI). Meanwhile, the features based on the frequency domain were the frequency median (FMD), frequency mean (FMN), modified frequency median (MFMD), modified frequency mean (MFMN), and frequency ratio (FR).

Equation (2) indicates the IEMG definition [42], where *n* is the batch size of the segmented data (64) and *X*_*i*_ represents *i*^th^ data in the dataset. The IEMG is the sum of the absolute value of the EMG signal, which can be treated as a signal power estimator [38].

(2) $$\begin{array}{c} \text{IEMG}=\sum_{i=1}^{n}\left|X_{i}\right|. \end{array}$$

The MAV, MMAV1, and MMAV2 can be defined by equation (3) [43], equation (4), and equation (5) [44], respectively, where *w*_*i*_ is the *i*^th^ modified weight of the mean absolute value, which is an important characteristic of the sEMG signals that are based on the time domain.

(3) $$\begin{array}{c} \text{MAV}=\frac{1}{n}\sum_{i=1}^{n}\left|X_{i}\right|, \end{array}$$

(4) $$\begin{array}{c} \text{MMAV}1=\frac{1}{n}\sum_{i=1}^{n}w_{i}\left|X_{i}\right|, \end{array}$$

(5) $$\begin{array}{c} \text{MMAV}2=\frac{1}{n}\sum_{i=1}^{n}w_{i}\left|X_{i}\right|\\ w_{i}=\left\{\begin{array}{cc} 0.25n\leq i\leq 0.75n,\\ \frac{4i}{n}, & i<0.25n,\\ \frac{4\left(i-n\right)}{n}, & i>0.75n. \end{array}\right. \end{array}$$

The MAVS, which indicates the variation between two adjacent batches, can be correctly represented by equation (6) [38], where *k* represents the *k*^th^ batch in the dataset.

(6) $$\begin{array}{c} {\text{MAVS}}_{k}={\text{MAV}}_{k+1}-{\text{MAV}}_{k}. \end{array}$$

The RMS can be described by equation (7) [39]. This quantity is modeled as an amplitude-modulated Gaussian random process whose RMS is related to the constant force and nonfatigue contraction [38].

(7) $$\begin{array}{c} \text{RMS}=\sqrt{\frac{1}{n}\sum_{i=1}^{n}X_{i}^{2}}. \end{array}$$

The VAR can be expressed by equation (8) [42]. This quantity indicates the difference between the signals in the dataset.

(8) $$\begin{array}{c} \text{VAR}=\frac{1}{n}\sum_{i=1}^{n}{\left(X_{i}-\bar{X}\right)}^{2}. \end{array}$$

The WL is defined by equation (9). This value, which is the cumulative length of the waveform over a segment, is influenced by the waveform amplitude, frequency, and duration [43].

(9) $$\begin{array}{c} WL_{k}=\sum_{i=1}^{n-1}\left|X_{i+1}-X_{i}\right|. \end{array}$$

The threshold crossings (TCs) are defined as the instances of the recorded data that crosses a threshold value during one batch.

Equation (10) represents the WAMP [39], which is the cumulative length of the waveform over a segment. This quantity indicates the number of times that the difference of consecutive amplitudes exceeded a predetermined threshold, *ℓ*.

(10) $$\begin{array}{c} {\text{WAMP}}_{k}=\sum_{i=1}^{n-1}f\left(\left|X_{i}-X_{i+1}\right|\right),\\ f\left(x\right)=\left\{\begin{array}{cc} 1, & x>\ell ,\\ 0, & \text{otherwise.} \end{array}\right. \end{array}$$

Equation (11) represents the SSI. This quantity is the cumulative length of the waveform over a segment. It also represents the accumulation of the bathed data power [38].

(11) $$\begin{array}{c} {\text{SSI}}_{k}=\sum_{i=1}^{n}\left(X_{i}^{2}\right). \end{array}$$

Equations (12) and (13) indicate the FMN [38] and FMD [44], respectively. These quantities use FFT to calculate some properties regarding the power spectrum density (PSD). However, the Pwelch values must be obtained for the calculation of the PSD in MATLAB. This is a difficult task to be executed using an MCU, as similar results are difficult to be obtained. Hence, in this study, we obtained a resemblance [45] between the Pwelch method and the PSD calculated using FFT through equations (14) and (15), respectively. This procedure was added to the MCU using the built-in FFT library from the STM32 DSP.

(12) $$\begin{array}{c} \text{FMN}=\frac{\sum_{i=1}^{n}f_{i}{\text{PSD}}_{i}}{\sum_{i=1}^{n}{\text{PSD}}_{i}}, \end{array}$$

(13) $$\begin{array}{c} \text{FMD}=\frac{1}{2}\sum_{i=1}^{n}{\text{PSD}}_{i}, \end{array}$$

(14) $$\begin{array}{c} \text{Pwelch}=2{\left(\left|fft\left(X_{i}\right)\right|\right)}^{2}, \end{array}$$

(15) $$\begin{array}{c} \text{PSD}={\left(\left|fft\left(X_{i}\right)\right|\right)}^{2}. \end{array}$$

The MFMN and MFMD were proposed by Phinyomark et al. [44]. MFMN is calculated as the sum of the product of the amplitude spectrum and frequency divided by the sum of the spectral intensity. MFMD is defined as half of the sum of the amplitude spectrum [38]. As a result, the amplitude spectrum of the signal can result in a volatile FFT.

The frequency ratio (FR) [46] is calculated in equation (16), where *fft*_max_ and *fft*_min_, respectively, represent the maximum and minimum values of the dataset after the fast Fourier transformation.

(16) $$\begin{array}{c} \text{FR}=\frac{fft_{\min}}{fft_{\max}}. \end{array}$$

The flag label (FL) shown in equation (17) indicates the decision after evaluating the received data batch. When the dataset includes more than three sampled data points that are labeled, the entire batch is considered for the demand of the decision to trigger the actuator. This feature was omitted in practical scenarios, and it is only available for real-time calibration of the neural network classifier.

(17) $$\begin{array}{c} \text{FL}=\left\{\begin{array}{c} 0,\;f<3,\\ 1,\;f\geq 3. \end{array}\right. \end{array}$$

The feature extraction was first built using MATLAB2019a considering a raw dataset stored in txt files. Each file contained more than 15000 samples of data. Sixteen feature extractions were applied for each channel of the sEMG signal, resulting in 32 features and one labeling data. These data were stored in csv files and were used, thereafter, in the classification stage.

After the offline data training procedure, the feature extracting model was coded again using the C language and downloaded into the MCU. The FFT was obtained by using the ARM_math and ARM_cFFT_Radix4 libraries [47]. 32 features were extracted from the two input channels. The output of the feature extraction was validated using a COM helper application and a JLINK debugger.

## 8. Classification

Many classification methods, such as k-nearest neighbours (k-NN) [26, 28], linear discriminant analysis (LDA) [26, 39], quadratic discriminant analysis (QDA) [28], support vector machine (SVM) [27, 28, 41], random tree (RT) [28], random forest (RF) [28, 41], artificial neural networks (ANN) [26, 38, 41], Bayes classifier [26, 38], self-organising map (SOP), and fuzzy classifiers [41], are available in the literature.

The Softmax classifier has outstanding performance when treating a multiclassification problem, as all types of features are normalized according to the number of classes. Furthermore, this classifier can clarify positive features [27]. In the binary classification problem in this study, the device is required to distinguish the triggering signal from the background noise, as the same triggering gesture pattern is used for the masking and unmasking actions. In this case, a Softmax classifier is adequate to solve this problem, as it yields fewer parameters than that of the other classifiers, owing to its simplicity. A large number of parameters would slow the computation speed and consume much flash memory of the MCU. In addition, the increase in complexity of the neural network results in the increase in difficulty to rewrite the model on a portable device.

We constructed the binary Softmax classifier using the 2.3.1 framework backend on TensorFlow 1.13.1. The IDE program on which the algorithm was developed was Pycharm 2020.3–Python version 3.7. No GPU was required, as the network structure and data type were not complicated.

For dataset recording, the person that tested the device was placed in a comfortable position and the electrode was firmly attached to the selected zygomaticus and bicipital muscles. A series of random movements of the limbs and changes in the countenance were performed while periodically executing the triggering pattern (simultaneous contraction of the zygomaticus and bicipital muscles). Whenever the targeting pattern was executed, the subject was requested to press the push button at the same time that he labels the corresponding data batch.

Throughout the offline model training stage, the features were extracted using MATLAB and stored in csv files, which were, thereafter, used in the training of the neural network. However, during the real-time optimization of the model, the features were directly extracted by the portable data processing unit and sent to the PC using UART. These data were again stored in txt files, which were, thereafter, converted into csv files for calibration. As a result, a more realistic dataset was acquired, and the Softmax classifier could be calibrated to achieve its best performance.

The accessed data were shuffled and, thereafter, divided into a training dataset and the test dataset using the K-fold method from the sklearn library. Meanwhile, the label value was converted into a one-hot code using the built-in function of Keras.

The structure of the constructed binary Softmax classifier is shown in Figure 11. Overall, the classifier was composed of one input layer, one hidden dense layer, and one output layer. The input layer had a 1 × 32 input dimension and received a flattened array of 32 features related to the bichannel sEMG input, which could be fed to the network in single frames or catches. The hidden dense layer of the classifier outputted an array of data size 1 × 64. A drop-out method, whose ratio was 0.02, was introduced to the network to perform a regularization task, preventing the overfitting of the classifier. The output dimension of the network was the same as the class number (2).

For the neural network training process, 40 epochs of 50 batches for each step were implemented. A categorical loss function was used for the loss assessment. The Adam algorithm was implemented for optimization.

The performance analysis of the classifier is shown in Figure 12.  Figure 12(a) shows the training and validation accuracy of the network. The average accuracy of 97.7% was achieved, and no significant difference was noticeable between the accuracies of the training and validation models, indicating that no overfitting or owe fitting occurred.  Figure 12(b) displays the loss of the network during the training and test stages. Both losses converge to a single value.

The weights and biases of the trained model were, afterward, converted into array metrics. The copied network of the Softmax classifier was reconstructed using the C language, and the parameters were included. The resulting neural network was repeatedly calibrated considering real-time features sent from the MCU, which were updated to increase the accuracy.

Nevertheless, not all 16 features used in this study should be used during real clinical applications. The FMN shows no significant variation during the test, while the variation of the other features was noticeable. Accordingly, some of the 15 discussed features should be changed in clinical applications.

## 9. Experiment and Results

Based on the mechanical structure 3D printed and real-time models downloaded, a functioning prototype of the proposed device was built, as indicated in Figure 13.

The mechanism and circuitry of the device were welted on a 5 mm acrylic board using hot-melt adhesives. Actuation of the mechanism was accomplished using a pair of FUTABA S3003 servo motors. Two sets of 5 V batteries were affixed on the board due to the connection plugin shape variance. In the left corner of Figure 13(c), the JLink device, CH340 UART module, and push button were detached using the portable device. The white ropes shown in Figure 13 were used to fasten the device to the subject.

To test the accuracy of the actual prototype, the accuracy was defined by [26]

(18) $$\begin{array}{c} \text{ACC}=\frac{T_{p}}{T_{p}+F_{N}+F_{P}}\times 100\%, \end{array}$$

where *T*_*P*_, *F*_*P*_, and *F*_*N*_ denote the number of correct recognitions, incorrect recognitions, and missed gestures. The subject wore the portable device for 1 min. The results are listed in Table 3.

Five tests were conducted considering a recording length of 1 min. Their overall average accuracy was 95.3%. During the test, the subject was asked to perform daily actions, such as drinking or walking, to simulate casual activities. The total number of gestures was not confined; therefore, the experiment could simulate casual activities within a fixed time interval. Based on the test results, therefore, the proposed portable face-shielding device was suitable for further implementation.

## 10. Conclusion

A portable face-shielding device utilizing sEMG was proposed, assembled, and proven to be feasible. The purpose of this research was to help disabled and paralyzed patients to independently wear face shields, reducing the risk of contamination due to the direct touch inside the face shield by the hands of ordinary people. Furthermore, new electrode materials using CNT/PDMS were proposed and tested to evaluate their dermotropic properties and electrical conductivity. The proposed device shows promising prospects for future implementation during the COVID-19 pandemic. Further product transitions are encouraged to target wear suitability and audience generalization.

## Figures and Tables

**Figure 1:** Data flow chart of the proposed device.

**Figure 2:** Research methodology diagram.

**Figure 3:** Experiment setups for feature extraction and classification model training.

**Figure 4:** Simplified model of the device. (a) Simplification of the motion form. (b) Parallelogram configuration of the four-bar linkage.

**Figure 5:** Simulations of the device in SOLIDWORKS. (a) 3D mechanism of the face-shielding device, including two equal four-bar linkages, two bases, and two connecting axles. (b) Optimized mechanism containing connectors and new supporting bases.

**Figure 6:** Design of CNT/PDMS composite electrodes.

**Figure 7:** Sample of CNT/PDMS electrode.

**Figure 8:** Electrode placement illustration.

**Figure 9:** Muscle selection and electrodes placement. (a) Positioning of the electrode on zygomaticus. (b) Electrode positioning on the bicipital muscle of the arm.

**Figure 10:** Raw data sent from the MCU to PC.

**Figure 11:** Neural network structure.

**Figure 12:** Assessment of the Softmax classifier. (a) Training and validation accuracy of the network. (b) Training and testing loss of the network.

**Figure 13:** Test pictures of the prototype. (a) Unshielded status of the device. (b) Shielded status of the device. (c) Assembled device prototype.

**Table 1:** Resistance comparison.

Ag/AgCl electrodes	CNT/PDMS electrodes
600∼800 Ω	200∼300 Ω

**Table 2:** CNT/PDMS electrodes parameters.

Total size	Conductive diameter (mm)	Thickness (mm)	Doping quality
Length 36.5 mm, width 30.2 mm	10	2	Less than 1 g

**Table 3:** Test result.

Number	*T*_*P*_	*F*_*N*_	*F*_*P*_	ACC (%)
1	29	0	4	87.9
2	23	0	1	95.8
3	22	0	0	100
4	40	0	0	100
5	38	1	2	92.7

## Data Availability

The raw/processed data and program source code required to reproduce these findings are as follows: https://github.com/JasonLvernex/BMI_automatics-faceshielding-device.
